# A Modified Quasisteady Aerodynamic Model for a Sub-100 mg Insect-Inspired Flapping-Wing Robot

**DOI:** 10.1155/2020/8850036

**Published:** 2020-12-22

**Authors:** Chenyang Wang, Weiping Zhang, Junqi Hu, Jiaxin Zhao, Yang Zou

**Affiliations:** National Key Laboratory of Science and Technology on Micro/Nano Fabrication, School of Electronic Information and Electrical Engineering, Shanghai Jiao Tong University, Shanghai 200240, China

## Abstract

This study proposes a modified quasisteady aerodynamic model for the sub-100-milligram insect-inspired flapping-wing robot presented by the authors in a previous paper. The model, which is based on blade-element theory, considers the aerodynamic mechanisms of circulation, dissipation, and added-mass, as well as the inertial effect. The aerodynamic force and moment acting on the wing are calculated based on the two-degree-of-freedom (2-DOF) wing kinematics of flapping and rotating. In order to validate the model, we used a binocular high-speed photography system and a customized lift measurement system to perform simultaneous measurements of the wing kinematics and the lift of the robot under different input voltages. The results of these measurements were all in close agreement with the estimates generated by the proposed model. In addition, based on the model, this study analyzes the 2-DOF flapping-wing dynamics of the robot and provides an estimate of the passive rotation—the main factor in generating lift—from the measured flapping kinematics. The analysis also reveals that the calculated rotating kinematics of the wing under different input voltages accord well with the measured rotating kinematics. We expect that the model presented here will be useful in developing a control strategy for our sub-100 mg insect-inspired flapping-wing robot.

## 1. Introduction

For decades, researchers have been interested in exploring the flapping mechanism of insects and developing insect-inspired flapping-wing micro air vehicles (FMAVs) [1–9]. In [6], we presented the world's smallest electromagnetically driven flapping-wing robot capable of liftoff, shown in Figure 1. To further develop the control strategy of the robot, its flapping aerodynamics must be analyzed and modeled.

The flapping flight of insects is characterized by a high angle of attack and a high rotational component, causing a large number of separations of the boundary layer and potentially generating vortices attached to the leading and trailing edges of the wings. These complex boundary conditions make it difficult to build an accurate steady aerodynamic model. Instead, researchers have attempted to develop quasisteady or unsteady aerodynamic models both for the flapping flight of insects and for insect-inspired robots [10–21]. For example, by studying a dynamically scaled model of the fruit fly (*Drosophila melanogaster*) [10], Dickinson et al. identify three mechanisms—delayed stall, rotational circulation, and wake capture—to explain how insects produce high lift at low Reynolds numbers. In a subsequent study, Sane and Dickinson [11] use blade element theory (BET) to develop a quasisteady aerodynamic model for insect flapping. From studies of free-falling cards [22–24], Bergou et al. [12] propose a 2-DOF quasisteady aerodynamic model for insect flapping that considers the circulation, dissipation, added mass, and inertial effect. In recent years, several improved models have been presented. For example, Nabawy and Crowther [16] propose a quasisteady aerodynamic model for the evaluation of the steady translational force coefficients of flapping wings in normal hover. The model is generic in that it can be applied to wings of arbitrary morphology and kinematics without the use of experimental data, and the aerodynamic components of the model are linked directly to morphology and kinematics via physical relationships. On this basis, Nabawy and Crowthe [17] propose a novel lifting-line theory introducing the concept of the equivalent angle of attack, which enables the capture of the steady nonlinear aerodynamics at high angles of attack and allows accurate estimation of aerodynamic forces from geometry and kinematic information alone. For detailed studies of the aerodynamic moment and the movement of the center of pressure on an insect wing, Han et al. [18] present an improved quasisteady aerodynamic model of a hawkmoth-scale flapping wing that considers the movement of the center of pressure. They find that the model becomes more suitable when the center of pressure is assumed to be at the half-chord rather than the quarter-chord. Nakata et al. [19] propose a novel CFD-informed quasisteady model which assumes that the aerodynamic forces on a flapping wing can be decomposed into quasisteady forces and parameterized based on CFD results and which is capable of predicting flapping-wing aerodynamic forces and power with higher accuracy. Lee et al. [20] present an improved quasisteady aerodynamic force and power model for rigid flapping by considering the effects of Reynolds numbers, Rossby numbers, wing aspect ratios, and taper ratios. Their model has the advantage of being applicable over a wider range of flow conditions without prior tuning or calibration. Wang et al. [21] propose a predictive quasisteady model by considering the wing's translation, rotation, and coupling, as well as the added-mass effect. This model shows high accuracy in predicting the center of pressure, the aerodynamic loads, and the passive pitching motion for various Reynolds numbers without any empirical parameters.

Based on the nonrigid connection of a flexible hinge, the artificial wing used in the robot we designed generates lift through its passive rotation while flapping. The kinematics of the wing can be considered as 2-DOF of flapping and rotating. In addition, since the observed deformation of the wing during flapping is negligible, it can be regarded as a rigid plate, similar to the approximation of a two-dimensional rigid plate (or wing) in Wang et al. [12, 23]. However, the latter assumes that the axis of rotation of the plate is on its midline and that the chord length is maintained—characteristics not found in insect wings or in insect-inspired robots.

The purpose of the present study is to provide a more accurate estimate of the lift and passive rotation generated by the robot's artificial wing. We first develop a quasisteady aerodynamic model based on BET by modifying the terms of dissipation and added-mass from [12]. We then report the findings of experiments performed to assess the model. The wing kinematics and the lift generated by the robot were captured simultaneously by a binocular high-speed photography system and a customized lift measurement system, respectively. The lift and passive rotation were calculated both on the basis of the model and from the experimentally captured wing kinematics under different input voltages. The results predicted by our model are in close accord with the experimental measurements.

## 2. Description of the Artificial Wing

### 2.1. Morphology

The artificial wing studied in this paper is morphologically similar to the *Eristalis tenax* wing [25], as shown in Figure 2.

To reduce the complexity of the artificial wing, the wing root, veins, and thickness of the insect wing are ignored. The plane profile and the geometric parameters of the artificial wing are shown in Figure 3.

The *x*_*w*_-axis and *y*_*w*_-axis represent the span and chord direction of the wing, respectively, and the direction of the *z*_*w*_-axis corresponds to the right-hand rule. *R* is the length of the wing (measured as 13 mm). *x*_*r*_ is the distance from the wing root of the wing *O*′ to the center of rotation *O*, which is small compared to *R* and is taken to be 0 in this paper. The green part shown in Figure 3 is the spanwise strip of the wing, *r* is the distance from the spanwise strip to the root of the wing, $\hat{r}=r/R$ is defined as the normalized distance, *d*_*r*_ is the width of the spanwise strip, and *d*_*y*_ is the width of a chord element on the spanwise strip. *P*_com_ is the center of mass of the wing, *P*_cog_ is the geometric center of the wing, *P*_*A*_ is any point on the spanwise strip, *P*_*M*_ is the midpoint of the spanwise strip, and *P*_*r*_ is the intersection of the spanwise strip and the *x*_*w*_-axis. The leading edge *y*_*l*_ and the trailing edge *y*_*t*_ of the wing are parameterized into functions of *y*_*l*_(*r*) and *y*_*t*_(*r*), respectively, as shown in Table 1, in which the coefficients are obtained by polynomial fitting of the morphology of the *Eristalis tenax* wing in [25] based on MATLAB (MathWorks Inc.).

The chord length *c* can then be expressed as *c*(*r*) = *y*_*l*_(*r*) − *y*_*t*_(*r*), and the area of the single wing can be integrated as *S* = ∫_0_^*R*^*c*(*r*)*dr* (calculated as 49.27 mm^2^). The mean chord is $\bar{c}=S/R$ (calculated as 3.79 mm), the normalized chord is defined as $\hat{c}=c/\bar{c}$, and the aspect ratio is $AR=R/\bar{c}$ (calculated as 3.43). A nondimensional radius of the *k*th moment of the wing area can then be expressed as ${\hat{r}}_{k}^{k}\left(S\right)=\int_{0}^{1}\hat{c}{\overset{\wedge }{r}}^{k}\text{d}\hat{r}$, as outlined in [25].  Table 2 compares the morphological parameters of the artificial wing and the *Eristalis tenax* wing.

### 2.2. Kinematics

The coordinate systems and the angles in 3-DOF of a wing are defined in Figure 4. The *x*_3_*y*_3_*z*_3_-coordinate system is defined as the experimental reference coordinate system, in which the *x*_3_*z*_3_-plane is the flapping stroke plane and the *y*_3_-axis is parallel to the average lift of the robot while hovering. The *x*_*w*_*y*_*w*_*z*_*w*_-coordinate system is defined to describe the fixed-wing plane. The flapping angle *φ* is defined as the opposite number of the rotation angle of the *x*_2_*y*_2_*z*_2_-coordinate system relative to the *x*_3_*y*_3_*z*_3_-coordinate system along the −*y*_3_-axis. The deviation angle *θ* is defined as the rotation angle of the *x*_1_*y*_1_*z*_1_-coordinate system relative to the *x*_2_*y*_2_*z*_2_-coordinate system along the *z*_2_-axis. The rotation angle *ψ* is defined as the rotation angle of the *x*_*w*_*y*_*w*_*z*_*w*_-coordinate system relative to the *x*_1_*y*_1_*z*_1_-coordinate system along the *x*_1_-axis. The directions of *φ*, *θ*, and *ψ* coincide with the directions of the *y*_3_-, *z*_2_-, and *x*_1_-axes, respectively. It is worth noting that the coordinate systems in Figure 4 are slightly offset for greater intuitiveness. In fact, all the coordinate systems share the same zero-point *O*.

It has been observed that there is hardly any deviation of the wing while flapping. Therefore, we assume in this study that *θ* ≡ 0. This means that the *x*_1_*y*_1_*z*_1_-coordinate system and the *x*_2_*y*_2_*z*_2_-coordinate system are completely coincident, so that only the flapping and rotating (2-DOF) kinematics of the wing need to be considered. In the following discussion, ^*i*^[·] represents the physical quantities in the *x_i_y_i_z_i_* coordinate system. _**i**_^**j**^**R** represents the coordinate transformation matrix of the *x*_*i*_*y*_*i*_*z*_*i*_*-*coordinate system with respect to the *x*_*j*_*y*_*j*_*z*_*j*_-coordinate system, as follows:

(1) R2w=1000cosψsinψ0−sinψcosψ,R32=cosφ0−sinφ010sinφ0cosφ.

The angular velocity of the wing and the linear velocity of any point _ _^**w**^**P**_**A**_ = [*r* *y* 0]^*T*^ in the *x*_*w*_*y*_*w*_*z*_*w*_-coordinate system can be expressed as

(2) ω w=ωx wωy wωz w=ψ˙00+R0φ˙0=ψ˙φ˙cosψ−φ˙sinψ,2w

(3) vA=vA,x wvA,y wvA,z w=ω w×PA w=yφ˙sinψ−rφ˙sinψyψ˙−rφ˙cosψ, w

where $\dot{\varphi }$ and $\dot{\psi }$ are the first derivative with respect to time of *φ* and *ψ*, respectively. Note that the linear velocity of each spanwise strip along the *x*_*w*_-axis is ignored based on BET; that is, we assume _ _^*w*^*v*_*A*,*x*_ = 0. In the *x*_*w*_*y*_*w*_*z*_*w*_-coordinate system, the wing inertia matrix after ignoring the thickness of the wing can be expressed as

(4) Iw w=Ixx w−Ixy w0−Iyx wIyy w000Izz w,

where _ _^*w*^*I*_*zz*_ = _ _^*w*^*I*_*xx*_ + _ _^*w*^*I*_*yy*_ and _ _^*w*^*I*_*xy*_=_ _^*w*^*I*_*yx*_.

The mass of the single artificial wing (*m*_*w*_) is measured as 0.5 mg, and the mass distribution of the wing in the *x*_*w*_*y*_*w*_*z*_*w*_-coordinate system is calculated by Inventor (Autodesk Inc.) as shown in Table 3, in which ^**w**^**P**_**com**_ is the center of mass of the wing.

## 3. Modeling Based on BET

In this section, the circulation, dissipation, added mass, and inertial effect are considered in the development of a quasisteady aerodynamics model based on BET.

### 3.1. Circulation

As shown in Figure 5, ^**w**^**P**_**M**_ is the midpoint of the spanwise strip, and ^**w**^**v**_**M**_ is the linear velocity at point *P*_*M*_ yielded by Equation (3). Utilizing the computational fluid dynamics (CFD) and experimental results of Pesavento and Wang [22], the aerodynamic force and aerodynamic moment generated by the circulation mechanism on a single spanwise strip can be expressed as

(5) dFcir w=ρairΓvM,x w−vM,y wvM,z wdr,dMcir w=PM w×dFcir w.

If *ρ*_air_ is the air density (taken as 1.29 × 10^−6^ g/mm^3^), _ _^*w*^*v*_*M*,*x*_ = 0, and Γ is the circulation, composed of the translational Γ_trans_ and rotational Γ_rot_ circulation,

(6) Γ=−12CTcvM wsin2α⏟Γtrans+12CRc2ψ˙⏟Γrot,

where *C*_*T*_ and *C*_*R*_ are dimensionless coefficients, respectively, taken as 1.8 and *π* [15, 22], and *α* = arccos (^*w*^*v*_*M*,*z*_/|^**w**^**v**_**M**_∣) is the angle of attack, defined as the angle between ^**w**^**v**_**M**_ and the *y*_*w*_-axis of each spanwise strip. Note that since the angle of attack of each spanwise strip is different, the angle of attack is defined for each strip rather than for the entire wing.

### 3.2. Dissipation

Based on [24, 26], for a chord element *d*_*y*_*d*_*r*_ on the spanwise strip shown in Figure 3, the aerodynamic force generated by the dissipation mechanism can be expressed as

(7) δFd w=0δFd,y wδFd,z w=−12ρairCDdydr0vA,y wvA,z2vA w wvA,z3 wvA w,

where the dimensionless coefficient *C*_*D*_ is taken as 3.4. The aerodynamic force and aerodynamic moment generated by the dissipation mechanism on a single spanwise strip can then be integrated as

(8) dFd w=∫ytylδFd w,dMd w=∫ytylPA w×δFd w.

### 3.3. Added Mass

During wing flapping, the acceleration and deceleration of the wing cause the surrounding air to accelerate and decelerate. In this process, the surrounding air pushes against the wings, creating the added-mass effect. For the translation and rotation of thin two-dimensional rigid wings, the aerodynamic force and aerodynamic moment generated by the added-mass effect on a single spanwise strip can be expressed (based on [27]) as

(9) dFadd w=00dFadd,z w=00−λzv˙r,z w+λzωω˙x wdr,dMadd w=dFadd,x wdFadd,y w0=−λzωv˙r,z w+λωω˙x wdrλzv˙r,z w+λzωω˙x wrdr0,

where v˙r,i w and ω˙x w are the first derivatives with respect to time of the linear velocity _ _^*w*^*v*_*r*_ of _ _^*w*^*P*_*r*_ and of _ _^*w*^*ω*_*r*_ in the *x*_*w*_*y*_*w*_*z*_*w*_-coordinate system, respectively. *λ*_*i*_ and *λ*_*ij*_ are the added-mass coefficients, defined as

(10) $$\begin{array}{c} \lambda_{z}=\frac{1}{4}\pi \rho_{\text{air}}c^{2},\\ \lambda_{z\omega }=\frac{1}{8}\pi \rho_{\text{air}}c^{2}\left(y_{l}+y_{t}\right),\\ \lambda_{\omega }=\frac{1}{16}\pi \rho_{\text{air}}c^{2}{\left(y_{l}+y_{t}\right)}^{2}+\frac{1}{128}\pi \rho_{\text{air}}c^{4}. \end{array}$$

### 3.4. Inertial Effect

Part of the aerodynamic force and moment generated by the wing is used for the linear and rotational acceleration of the wing itself. Although the mass of the wing is small, its inertial effect is not negligible. In the *x*_*w*_*y*_*w*_*z*_*w*_-coordinate system, the inertial force and the inertial moment of a single wing can be expressed as

(11) Finertia w=Finertia,x wFinertia,y wFinertia,z w=−mwv˙com w,Minertia w=Minertia,x wMinertia,y wMinertia,z w=−Iw wω˙ w,

where v˙com w is the first derivative with respect to time of the linear velocity _ _^**w**^**v**_**com**_ of _ _^**w**^**P**_**com**_ in the *x*_*w*_*y*_*w*_*z*_*w*_-coordinate system.

### 3.5. Total Aerodynamic Force and Moment

From the above, the total aerodynamic force and the total aerodynamic moment acting on a single wing can be integrated in the *x*_*w*_*y*_*w*_*z*_*w*_-coordinate system as

(12) FAero w=FAero,x wFAero,y wFAero,z w=∫0RdFcir w+dFd w+dFadd w+Finertia w,

(13) MAero w=MAero,x wMAero,y wMAero,z w=∫0RdMcir w+dMd w+dMadd w+Minertia w.

It is clear from this that the aerodynamic force and moment are completely determined in the proposed model by the morphology and 2-DOF transient kinematics (*φ* and *ψ*) of the artificial wing. In addition, some unsteady aerodynamic mechanisms, such as the start-up vortices [28], the spanwise flow [29], the wake capture [10], and the tip vortices [30], are partly included in the dimensionless aerodynamic coefficients used in this study. In this way, the aerodynamics generated by some unsteady-state mechanisms are also accounted for in the model.

## 4. Experiments and Analysis

### 4.1. Measurement of Wing Kinematics and Lift

With the fixed-shape artificial wing designed for our robot, the flapping aerodynamics are determined only by the 2-DOF wing kinematics of *φ* and *ψ*. However, the lift generated by the robot is also valuable in assessing the model. Our experiments measured the kinematics of the wing and the lift of the robot simultaneously. As illustrated in Figure 6(a), a binocular high-speed photography system was used to measure the flapping and rotational kinematics of the left wing of the robot. At the same time, the lift generated by the robot was measured using a customized lift measurement system described in [31] and illustrated in Figures 6(b) and 6(c). A trigger was used to ensure that the photography system and the lift measurement system worked synchronously.

More specifically, the binocular high-speed photography system consisted of two high-speed cameras (Phantom LC111, working synchronously at 3000 fps), with the tips and intersections of the wing veins serving as mark points. Based on the binocular ranging method and three-dimensional motion reconstruction, the spatial position of these mark points in each frame is obtained by the direct linear transformation (DLT) method [32], and the flapping and rotating kinematics are then derived from the geometric relationship of these mark points.

For the lift measurement, the robot is mounted vertically on the support plate of the lift measurement system, as shown in Figure 6(c). The real-time lift generated by the robot is transformed by the deformable Invar-made double-cantilever beam into a slight displacement in the vertical direction of the target plate, and the real-time lift of the robot is then extracted by measuring the real-time displacement of the target plate using a capacitive displacement sensor (CS005, Micro-Epsilon). Since a magnet is used as part of the electromagnetic actuator in the robot, a long truss made of carbon fiber was introduced to extend the distance between the robot and the Invar-made support plate so as to prevent electromagnetic interference. After calibration, the lift measurement system had a dynamic resolution of 0.457 *μ*N (0.82 mg), and a sensitivity of 2.19 *μ*m/mN.

The sub-100 mg insect-inspired flapping-wing robot presented in [6] was used as the prototype for the measurement. Sinusoidal voltages with a fixed frequency of 80 Hz were applied to the robot. The measured flapping kinematics *φ*_meas_ and rotating kinematics *ψ*_meas_ of the left wing under different voltage amplitudes are shown in Figures 7(a) and 7(b), in which each curve is obtained from these measurement points by sixth-order Fourier fitting. The rotating kinematics are delayed overall with respect to the flapping kinematics by a quarter of a stroke cycle. As the amplitude of the input voltage is increased, the flapping and rotating kinematics of the wing change more dramatically. The relationship between the peak-to-peak amplitude of the measured wing kinematics and the input voltage amplitude is shown in Figure 7(c). It is clear that the amplitudes of the wing kinematics can be modulated by the input voltage amplitude, which is helpful in controlling the lift of the robot.

### 4.2. Calculated Aerodynamics

By substituting the morphology shown in Table 1 and the measured flapping and rotating kinematics of the wing into Equations (12) and (13), the aerodynamics of the single artificial wing under different input voltage amplitudes were calculated based on the proposed quasisteady aerodynamic model, as shown in Figure 8. Obviously, the magnitudes of the aerodynamic force and moment are determined by the amplitude of the input voltage. For the calculated aerodynamic force _ _^3^*F*_Aero,*y*_ along the *y*_3_-axis (i.e., the lift direction of the robot while hovering), the total force and circulation force almost coincide, indicating that the circulation mechanism makes the dominant contribution to the aerodynamic force. The two peaks of the total aerodynamic force are located in the middle of the upstroke and the middle of the downstroke, with the translational circulation force making the main contribution. However, at the reversal of the stroke, the total aerodynamic force is close to zero or even negative. Note that the curve should be symmetric around the stroke reversal; the difference between the two peaks of force shown in Figure 8 is mainly due to the asymmetry of the wing kinematics caused by assembly and measurement errors. Since the flapping frequency of the robot is 80 Hz, the mean aerodynamic force is more valuable for flight control than the transient force. The distribution of the mean aerodynamic force after cycle averaging is shown in Table 4. The mean force is almost entirely determined by the circulation and the added mass, while the contributions of the dissipation and the inertial effect are negligible. Unlike the aerodynamic force, the calculated aerodynamic moment is mainly determined by the dissipation, the added mass, and the inertial effect rather than by the circulation. Since both the added-mass moment and the inertial moment are proportional to the linear and angular acceleration of segments of the wing at specific points, the trends of the added-mass moment and inertial moment are similar. Both the dissipation moment and the circulation moment are greater in the middle of the upstroke and downstroke, while they are almost zero at the reversal of the stroke.

### 4.3. Experimental Verification

To verify the applicability of our quasisteady aerodynamic model, we analyzed the lift and the passive rotation generated by the robot based both on the model and on experimental measurements.

#### 4.3.1. Lift Estimated by the Aerodynamic Force

The robot we designed consists of two wings, the kinematics of which are assumed to be perfectly s1ymmetric while hovering. Thus, the calculated lift generated by the robot can be expressed as

(14) Lcalc=2∙FAero,y 3.

To reduce the interference from mechanical and electrical noise at high frequencies, the measured instantaneous lift generated by the robot was filtered by a digital low-pass filter with a cutoff frequency of 300 Hz.  Figure 9 compares the measured and the calculated lift forces generated by the robot under different input voltages during one flapping cycle. The measured lift *L*_meas_ and the calculated lift *L*_calc_ are in good accord with regard to overall amplitude and trend, but unlike the calculated results, the measured amplitude of the upstroke is close to that of the downstroke. This indicates that the lift generated by the robot in the actual process is to some extent insensitive to the imperfect symmetry of the wing kinematics. Considering the unavoidable simplification in the mathematical model, the transient deviations between the measured and calculated results are acceptable. Both the measured curve and the theoretical curve show that the lift generated by the flapping wings fluctuates strongly, especially near the stroke reversal point, where the transient lift may even be negative.  Figure 9(e) compares the calculated mean lift ${\overset{¯}{L}}_{\text{calc}}$ to the measured mean lift ${\overset{¯}{L}}_{\text{meas}}$ of the robot under different input voltage amplitudes after cycle averaging. The comparison demonstrates the accuracy of the proposed quasisteady aerodynamic model in estimating the lift generated by the robot.

Although the values of the aerodynamic constants *C*_*T*_, *C*_*R*_, and *C*_*D*_ in the model are assumed from experience in our calculations, it is interesting to study the changes in the calculated lift of the robot when these three constants fluctuate separately. As described in Section 3, the total aerodynamic force acting on a single wing _ _^**w**^**F**_**Aero**_ is linear with *C*_*T*_, *C*_*R*_, and *C*_*D*_, respectively. With the fixed morphology and captured kinematics of the wing, the change in the mean lift of the robot is therefore directly proportional to the change in each aerodynamic constant. That is,

(15) $$\begin{array}{c} \Delta {\overset{¯}{L}}_{\text{calc}}\propto \Delta C_{i} \end{array}$$

where *C*_*i*_ refers to *C*_*T*_, *C*_*R*_, and *C*_*D*_, respectively. In order to quantify the relationship between the relative change in the mean lift of the robot and the relative change in each aerodynamic constant, we designate the sensitivity of the former to the latter as *k*_*i*_ (i.e., *k*_*T*_, *k*_*R*_, and *k*_*D*_, respectively). Then,

(16) $$\begin{array}{c} \frac{\Delta {\overset{¯}{L}}_{\text{calc}}}{{\overset{¯}{L}}_{0}}=k_{i}\frac{\Delta C_{i}}{C_{i0}}, \end{array}$$

where *C*_*i*0_ is the assumed value used in Section 3 ( *C*_*T*0_ = 1.8, *C*_*R*0_ = *π*, and *C*_*D*0_ = 3.4), and ${\overset{¯}{L}}_{0}$ is the calculated mean lift of the robot corresponding to *C*_*i*0_. Considering that the range of Δ*C*_*i*_/*C*_*i*0_ is [-30%, 30%], we now use the model to calculate the corresponding relative changes in the mean lift of the robot under the input voltages from 0.1 V to 1.1 V. For simplicity, Figure 10 shows just a part of the calculated results. The calculated *k*_*T*_ varies mostly between 0.55 and 0.65, which is 2-3 times the corresponding *k*_*R*_, while *k*_*D*_ is close to zero under any input voltage. These results indicate that changes in *C*_*T*_ and *C*_*R*_ are more likely to cause changes in the calculated mean lift and that changes in *C*_*D*_ have almost no effect on the lift. This finding is similar to the results illustrated in Figure 8 and Table 4; that is, the circulation (especially the translational circulation) is the dominant contributor to the calculated lift, while the contribution of the dissipation is negligible.

#### 4.3.2. Passive Rotation Estimated by the Aerodynamic Moment

As shown in Figure 2, each side of the artificial wing is connected to the transmission by a flexible hinge. Due to the nonrigid connection of the hinge, the flapping of the wing produces passive rotations, which are the main factor for the generation of lift [33, 34]. In this study, the rotating kinematics of the wing are accurately obtained by the binocular high-speed photography system based on three-dimensional motion reconstruction. However, further control tests of the robot require that the rotating kinematics of the wing be estimated quickly and easily rather than measured accurately. The binocular high-speed photography system requires at least two high-speed cameras as well as non-real-time image processing due to a large amount of data and therefore is more complex and less efficient than estimations generated by a mathematical model. The flapping kinematics of the wing can be easily measured in real time by only one high-speed camera. Based on the aerodynamic moment calculated using the model and on the measured flapping kinematics, we can analyze the 2-DOF dynamics of the robot and calculate the rotating kinematics. Since the artificial wings are considered to be rigid plates, the passive rotation of each wing is determined mainly by the aerodynamic moment (*M*_*A*_) acting on the entire wing, the gravity moment (*M*_*G*_) of the wing, and the torsional stiffness (*k*_*ψ*_) of the wing hinge. The gravity moment *M*_*G*_ is expressed as

(17) MG= wPcom w×R2w0−mwg0.

The wing hinge used in the robot is a sandwich structure consisting of a flexible polymer middle layer between thin, rigid outer layers, as shown in Figure 11. The torsional stiffness can be expressed as

(18) $$\begin{array}{c} k_{\psi }=\frac{E_{h}t_{h}^{3}w_{h}}{12l_{h}}, \end{array}$$

where *E*_*h*_ (3.5 GPa) is the elastic modulus of the flexible polymer layer and *l*_*h*_ (120 *μ*m), *w*_*h*_ (1800 *μ*m), and *t*_*h*_ (7.5 *μ*m) are, respectively, the length, width, and thickness of this layer.

From the analysis in Section 3, in the *x*_*w*_*y*_*w*_*z*_*w*_-coordinate system, the total moment that causes the passive rotation of the wing can be expressed as

(19) Mw w=Mw,x wMw,y wMw,z w=MA w+MG w+−kψψ00.

According to [35], the dynamics of the wing in 2-DOF (flapping and rotating) can be modeled as follows, based on the principle of virtual power:

(20) Mw w∙δω wδψ˙=0.

Substituting Equations (4), (13), and (19) into Equation (20) yields

(21) Ixxψ¨ w−Ixyφ¨cosψ−Ixxφ˙2sinψ w wcosψ−MA,x w−mwgycom wsinψ+kψψ=0,

where *^w^M_A,x_* is (in accordance with Equation (13)) solely a function of *φ* and *ψ* given the fixed morphology of the artificial wing. Therefore, by substituting the measured flapping kinematics *φ*_meas_ into Equation (21), the calculated rotating kinematics *ψ*_calc_ of the wing are obtained as shown in Figure 12. The measured rotating kinematics *ψ*_meas_ under the same input conditions are also plotted to verify the accuracy of the calculation results. It is clear that the calculated rotating kinematics *ψ*_calc_ are close to the measured results *ψ*_meas_ in terms of overall amplitude and trend, especially when the amplitude of the input voltage is relatively large. However, the amplitude of rotation is slightly overestimated by the proposed model at local positions such as the peaks in Figure 12, and the overestimation gradually increases as the input voltage (i.e., the amplitude of the flapping kinematics) decreases. The main reason is that when the flapping frequency is fixed and the flapping amplitude is reduced, the contribution of the translational aerodynamics to the drag force is further reduced due to the low flapping velocity. Furthermore, the passive rotation of the wing is slightly restricted by the unavoidable minor shaking and bending of the wings, and these unfavorable factors become significant as the flapping amplitude of the wings is further decreased. As a result, the accuracy of the model's estimation of the passive rotation declines with the decrease in the flapping amplitude. Like the lift results, the measured rotating kinematics are more symmetric about the stroke reversal point than the calculated rotating kinematics because the mathematical model is slightly sensitive to the asymmetry of input wing kinematics. Since the flapping amplitude of the robot is generally above ±55° in actual flight tests, and the model's estimates of the passive rotation in this range are relatively accurate, the estimations are a useful resource for the control of the robot.

## 5. Conclusion

In this paper, we present a modified quasisteady aerodynamic model for an electromagnetically driven sub-100-milligram insect-inspired flapping-wing robot whose design was presented in [6]. Based on the blade-element theory, the aerodynamic mechanisms of the circulation, dissipation, added mass, and inertial effect are considered in developing the model. Since the deviation of the artificial wing is negligible for our robot, the aerodynamics generated on the wing are completely determined, in this model, by the wing morphology and the 2-DOF wing kinematics of flapping and rotating.

To verify the applicability of the model, the wing kinematics and the lift generated by the robot were measured synchronously by a binocular high-speed photography system and a customized lift measurement system. Based on the measured flapping and rotating kinematics of the artificial wing, we calculated the aerodynamic forces and moments acting on the wing under different input voltages. Our results show that the circulation mechanism makes the dominant contribution to the transient aerodynamic lift, while the contributions of the dissipation and the inertial force are minimal. However, the aerodynamic moment is mainly determined by the dissipation, added mass, and inertial effect rather than by the circulation. Combined with the synchronous lift measurement of the robot, the transient lift and the mean lift estimated by the model are all in good agreement with the measured results under different input voltages. In addition, the robot generates lift by the passive rotation of the wings. Although the passive rotation can be captured by the binocular high-speed photography system used in this study, a more convenient way to estimate it is needed. To supply this need, we analyzed the 2-DOF flapping-wing dynamics of the robot based on the proposed model and obtained estimates of the rotating kinematics from the measured flapping kinematics alone. The calculated rotating kinematics of the wing under different input voltages are all in good accord with the measured values.

We therefore conclude that the modified quasisteady aerodynamic model developed in this study is applicable with high accuracy to the sub-100 mg insect-inspired flapping-wing robot presented previously and that the model will provide theoretical support for the development of control strategy.

## Figures and Tables

**Figure 1:** The sub-100 mg insect-inspired flapping-wing robot used as the prototype in this paper.

**Figure 2:** Shape of (a) the artificial wing and (b) the *Eristalis tenax* wing from [25].

**Figure 3:** The plane profile and the geometric parameters of the artificial wing.

**Figure 4:** Definitions of the coordinate systems and the kinematics of the left artificial wing.

**Figure 5:** A single spanwise is taken as an example to define the circulation and angle of attack. The angle of attack is the angle between the velocity of the midpoint and the *y*_*w*_-axis of the spanwise strip; it varies between −*π*/2 and *π*/2. The angle of attack in this case is negative.

**Figure 6:** (a) Setup of the lift measurement for the designed robot. (b) Photo of the measurement with two high-speed cameras. (c) Schematic of the customized lift measurement system.

**Figure 7:** The measured 2-DOF wing kinematics of (a) flapping and (b) rotating. For simplicity, measured results under only three input voltages are plotted, and each curve is obtained from the measured points by sixth-order Fourier fitting. Figure (c) shows the relationship between the peak-to-peak amplitude of the measured wing kinematics and the input voltage amplitude.

**Figure 8:** The aerodynamic force along the *y*_3_-axis _ _^3^*F*_Aero,*y*_ and moment along the *x*_*w*_-axis _ _^*w*^*M*_Aero,*x*_ under the input voltage amplitudes of (a) 1.1 V, (b) 0.8 V, and (c) 0.5 V.

**Figure 9:** The measured and calculated lift of the robot under the input voltage amplitudes of (a) 1.0 V, (b) 0.8 V, (c) 0.6 V, and (d) 0.4 V. (e) The relationship between the mean lift of the robot and the input voltage amplitude.

**Figure 10:** Analysis of the sensitivity of the calculated mean lift of the robot to the aerodynamic constants of *C*_*T*_, *C*_*R*_, and *C*_*D*_ under the input voltage amplitudes of (a) 1.0 V, (b) 0.8 V, (c) 0.6 V, and (d) 0.4 V (the number of input values is limited for simplicity).

**Figure 11:** Schematic of the flexible wing hinge.

**Figure 12:** The measured and calculated rotating kinematics of the artificial wing under the input voltage amplitudes of (a) 1.0 V, (b) 0.8 V, (c) 0.6 V, and (d) 0.4 V.

**Table 1:** The leading edge function and trailing edge function of the artificial wing.

Coefficients	*a*_1_	*a*_2_	*a*_3_	*a*_4_	*a*_5_	*a*_6_
*y*_*l*_	3.510*E* − 1	−1.428*E* − 1	4.537*E* − 2	−6.942*E* − 3	5.042*E* − 4	−1.430*E* − 5
*y*_*t*_	-4.442	1.941	−4.299*E* − 1	5.093*E* − 2	3.023*E* − 3	7.091*E* − 5
$y=\overset{6}{\underset{i=1}{\sum }}\left(a_{i}r^{i}\right)$						

**Table 2:** Morphological parameters of the artificial wing and the *Eristalis tenax* wing [25].

Parameters	Artificial	*Eristalis tenax*
*R* (mm)	13.0	11.4
Aspect ratio	3.43	3.58
*r*_1_(*S*)	0.474	0.471
*r*_2_(*S*)	0.534	0.534
*r*_3_(*S*)	0.579	0.579

**Table 3:** Mass distribution of the artificial wing.

^**w**^ **P**_**com**_ (mm)	(4.9481, -0.4927)
^*w*^ *I*_*xx*_ (mg·mm^2^)	1.196404184
^*w*^ *I*_*yy*_ (mg·mm^2^)	22.657024402
^*w*^ *I*_*xy*_ (mg·mm^2^)	-0.468631666

**Table 4:** Distribution of the mean aerodynamic force.

Input voltage	1.1 V	0.8 V	0.5 V
Total (mN)	4.22*E* − 1	2.07*E* − 1	7.33*E* − 2
Circulation (mN)	3.76*E* − 1	1.85*E* − 1	6.32*E* − 2
Dissipation (mN)	−9.83*E* − 6	−3.34*E* − 4	1.93*E* − 5
Added mass (mN)	4.54*E* − 2	2.19*E* − 2	1.00*E* − 2
Inertial effect (mN)	−8.41*E* − 5	−8.12*E* − 5	−5.58*E* − 6

## Data Availability

The data used to support the findings of this study are available from the corresponding author upon request.
